The article "Family Exit and Firms' Investment Efficiency Based on Dynamic Changes: Evidence from Chinese Family Firms" was published in 2022. Journal: Comput Intell Neurosci.

# Family Exit and Firms' Investment Efficiency Based on Dynamic Changes: Evidence from Chinese Family Firms

**DOI:** 10.1155/2022/7572891

**Published:** 2022-07-31

**Authors:** Tengyan Wang, Qiaoling Peng, Haiyan Song

**Affiliations:** ^1^Faculty of Professional Finance & Accountancy, Shanghai Business School, Shanghai, China; ^2^School of Economics and Management, Shanghai Maritime University, Shanghai, China; ^3^School of Finance, University of International Business and Economics, Beijing, China

## Abstract

This study provides evidence about the influence of family exit on firms' investment efficiency using a sample of 6,842 firm-year observations of Chinese family (and family-exiting) firms from 2003 to 2019. Based on panel data, we find that family exit has negative effects on firms' investment efficiency. Further analysis also indicates that family exit can decrease firms' investment efficiency under low investment levels and increase their investment efficiency under high investment levels. We test the market reaction when family members are punished by the SEC and find that the market's reaction is significantly negative, which implies that the capital market cares about family managers and controllers.

## 1. Introduction

Worldwide, family firms are a unique business group that contributes to economic growth and activities, especially in China [1]. With the development of the economic reform and opening up in China, the first generations of family firms are becoming increasingly older. Thus, these family firms are facing the urgent problem of a succession plan, that is, who will inherit the firm and how will oversight of the firm be passed on. Generally, most families would like to transfer the family firm to their children. However, there are many problems in the transfer process. The one-child policy caused families to have only one child, increasing the risk in family firms' succession plans. If the only child does not wish to take over the firm or has no management ability, then the firm has no choice but to be transferred to someone outside the family. The other situation is that when the family cannot bypass internal and external roadblocks, it will not be able to continue to be the majority shareholder. When there is no one to inherit the firm, there are two main options for a family to choose from. One is hiring nonfamily members to manage the firm, and the other choice is selling the firm to others. Will the firm benefit when the family exits? This study analyses the problem from the perspective of investment efficiency.

According to traditional finance theory, investment efficiency is defined as the undertaking of projects with a positive net present value [2]. Investment in good capital projects brings additional value to the firm, and it is rational to pursue as many value-maximizing investment opportunities as available [3]. Firms' investment efficiency is a type of measurement of firm performance [4, 5]. Investment efficiency is one of the important aspects of the difference between the performance of family and nonfamily firms. In this study, we focus on firms in which family members exit to determine the effect of decreasing family involvement on firms' investment efficiency and situations in which family firms obtain better investment performance. In this paper, we use the model in Richardson [6] to measure firms' investment efficiency.

Many factors affect a family firm's inheritance. If the family cannot choose a suitable person to inherit the firm, family exit may be a better choice [7]. The literature has revealed the difference between family and nonfamily firms. Family firms may be better or worse than nonfamily firms because there are two types of family firms [4]. However, the dynamic effect of family firms is not clear. Our study focuses on the dynamic change in family firms to determine the effect of family exit on the investment efficiency of Chinese family firms. More specifically, this study aims to provide empirical evidence to answer the following questions: does family exit influence firms' investment efficiency? What situation can help a family firm improve its performance?

To answer these questions, our study tests the effects of family exit on investment efficiency using Chinese listed family firms from 2003 to 2019. Based on the literature, we measure family exit in two ways. One way is from a managerial perspective: if a family firm hires nonfamily members as managers, we consider the firm to be a family-exiting firm. The other way is from the control power perspective: If the family gives up some of its shares to the extent that it is no longer the majority shareholder, we also consider the firm to be a family-exiting firm. Based on a difference-on-difference (DID) model, we find that family exit decreases investment efficiency. Moreover, we find a possible reason family exit decreases firms' investment efficiency.

To avoid the problem of endogeneity, we perform the DID analysis and inspect how lower family involvement affects firms' investment efficiency. Our results indicate that when family members give up management or control power, doing so decreases firms' investment efficiency. Furthermore, we test the importance of family members to family firms and find that the market reaction fluctuates severely if family members are punished by the SEC. In the analysis, we find different effects of family involvement on different firms' investment efficiency. Lower family involvement can improve a firm's investment efficiency when the firm's investment level is high, and vice versa.

Our study contributes to the literature in the following ways. First, it complements the growing body of literature investigating how family firms' behavior affects firm performance, especially investment efficiency. Second, this study contributes to the literature by conducting a dynamic analysis of change in family firms, whereas the previous literature mostly focused on the difference between family and nonfamily firms. Lastly, this study provides empirical evidence based on a transition economy, China, rather than developed countries.

## 2. Literature Review and Hypotheses

There are some studies on how to understand the difference between family and nonfamily firms [8–10], but there is abundant work on the ways in which family firms become nonfamily firms and the outcomes of doing so.

In recent years, the development of family business research has broadened beyond family members to study other actor groups working in family firms [11]. Some scholars believe that when family members exit from a family firm, doing so can increase the firm's innovation inputs and relieve financial constraints [12]. Regarding firms' investment efficiency, they have found that agency costs can have a negative effect on firms' best investment level, and management may also ignore investment efficiency to pursue the private benefits of controlling shareholders [13, 14].

Powerful family bonds can also exist outside the boundaries of the family firm and family business group, which can have valuable implications for the family firm itself [15]. From this perspective, nonfamily management may decrease firms' investment efficiency. First, managers from outside the family may wish to build a business empire for themselves. When building a business empire, managers may wish to overinvest [16]. They may also prefer to satisfy the firm's performance requirements and invest more than what the firm needs [3]. This selfish behavior can decrease a firm's investment efficiency. Second, nonfamily managers can boost a firm's short-term performance and then move to a new firm before it is revealed that the performance was a result of a short-term decision [17]. The short-term decision may decrease the firm's investment efficiency in the long term. Third, compared with family managers, nonfamily managers may wish to maintain higher cash holdings [6]. Therefore, nonfamily managers can invest less than family managers; hence, when family firms are run by nonfamily members, such leadership can lead to underinvestment, which easily decreases a firm's investment efficiency.

When family members influence a firm's management or control power level, their locality can reduce managers' myopia [18]. Moreover, the performance of a family firm is important to family managers [19]. Thus, family managers or controllers will try their best to improve the firm's performance, including ensuring investment efficiency [20]. From the perspective of the natural factor, family CEOs have fewer incentives to chase short-term gains. Family CEOs are from the family circle; thus, they face less pressure to demonstrate their ability [5]. Therefore, they prefer to increase the firm's investment efficiency from a long-term perspective. Moreover, they have a much longer horizon to balance short-term financial gains and long-term performance.

Investment decisions vary from company to company and are based on investment opportunities [2, 21]. Generally, the most appropriate investment decisions are made by managers who are the most familiar with the firm [22]. Compared with outsiders, family managers have intimate knowledge of the family firm, and they can make more appropriate investment decisions to achieve the firm's goals [23]. Moreover, a forecast of a family firm carried out by family members is more accurate, and a quality forecast increases firm-level investment efficiency.

Furthermore, when a family member is the chair of the board, such a situation integrates the reputation of the controlling family and the firm [20]. Family members also protect their reputation for more investor attention. Thus, they will wish to look for more investment opportunities and increase investment efficiency. Moreover, family members are important franchisors, which implies that the skills and resources that they provide to franchisees through strong relationships and training efforts are the foundation for capability development [23, 24]. Involving the family in the franchising business improves social relationships and knowledge sharing, which can increase investment efficiency.

There is evidence that pyramidal ownership improves investment efficiency, whereas cross-ownership weakens investment efficiency [25]. The ownership of most family firms is pyramidal, and a family firm's ownership style changes as family members exit the firm. When family members own a large proportion of the firm, family wealth is tied up with firm wealth, and the well-being of family owners closely depends on the success of the business [26]. Thus, family managers will try their best to increase the firm's investment efficiency to hold onto their family wealth.

## 3. Data and Research Methodology

### 3.1. Sample

Our initial data are from “Family Firm Research” in the CSMAR database and consist of family firms from 2003 to 2019. Some family firms disappeared from the database because of family exit; we manually compensate for these firms. After deleting missing values, we obtained 6,842 observations. We manually defined the family exit data, including 2,594 observations of firms that hired nonfamily managers and 122 observations of firms that gave up controlling power. The financial data are also from the CSMAR database; we exclude firms in the financial industry.

### 3.2. Methodology and Regression Models

Our study establishes a DID regression model to test the hypothesis.

(1) $$\begin{array}{c} \text{Investment }{\text{Efficiency}}_{i}=\beta_{0}+\beta_{1}\text{Transfer}\times \text{Post}+\beta_{2}{\text{Controls}}_{i}+\theta_{i}, \end{array}$$

where Post is an interblock dummy variable—family-exiting firms are the treatment group, and “nonfamily-exiting” firms are the control group. The observation in the control group takes the value of 0, and an observation in the treatment group takes the value of 1. The transfer is a time dummy variable; an observation before family exit takes the value of 0, and an observation after family exit takes the value of 1. Transfer × Post is an interaction variable of transfer and post. This interaction variable is the key variable in our study, showing the net effect of family exit on firms' investment efficiency. If the interaction variable is positive, family exit decreases firms' investment efficiency, and vice versa. To better analyze the relationship between family exit and firms' investment efficiency, all the regressions are performed using the DID model.

### 3.3. Measurement of Variables

#### 3.3.1. The Dependent Variable

Following previous studies [6], we measure investment efficiency as the residual of the model below. The larger the absolute value of the residual, the lower the investment efficiency of the firm.

(2) $$\begin{array}{c} {\text{Investment}}_{\text{tj}}=b_{0}+b_{1}\;{\text{Tob}}_{t-1,j}+b_{2}\;{\text{Lev}}_{t-1,j}+b_{3}\;{\text{Cas}}_{t-1,j}+b_{4}\;{\text{Age}}_{t-1,j}+b_{5}\;{\text{Siz}}_{t-1,j}+b_{6}\;{\text{Ret}}_{t-1,j}+b_{7}\;{\text{Investment}}_{t-1,j}+\varepsilon , \end{array}$$

where Investment denotes the firm's investment level, which we measure as the sum of fixed, intangible, and other long-term assets minus the cash flow from selling assets, divided by the previous year's assets. Tob is the firm's growth opportunity; Lev is the firm's leverage; Cas is the firm's cash holdings; Age is the firm's years since being listed; Siz is the firm's natural log of assets; and Ret is the firm's return in the year.

In the subsequent regression tests, the investment level is defined by the model. When the residual of the model is negative, the firm's investment level is considered low. Additionally, the firm's investment level is considered high when the residual of model (2) is positive.

#### 3.3.2. The Independent Variable

There are two paths by which a family exits a family firm. One is to hire a nonfamily manager, with the family still having the firm's control power. The other is partly or wholly selling the firm to others, meaning that the family will not control and manage the firm.

There is no consistent definition of family firms in the literature. Based on the previous literature and the aim of our research, we use two independent standards to define family firms [22, 27]. The first standard requires the family firm to satisfy the following: (1) the actual controller can be traced back to family members; (2) the majority shareholder is a family member; and (3) family members are CEOs or managers. If this type of family firm hires a nonfamily manager, we call it a family-exiting firm. When this type of family firm hires a nonfamily manager and the firm's control power is still in the hands of the family, we denote it as tra1, which takes the value of 1. In family members are still the managers, we denote it as transfer1, which takes the value of 0.

The second standard requires the family firm to satisfy the following: (1) the actual controller can be traced back to family members, and (2) the majority shareholder is a family member. If this type of family firm gives up the controlling power, we call it a family-exiting firm. When this type of family firm partly or wholly sells the firm to others, the family will not control and manage the firm; we denote this as tra2, which takes the value of 1. If the controlling power is still in the hands of family members, we denote it as tra2, which takes the value of 0.

#### 3.3.3. Adjustment Variables

  Marketization level. The variable means the extent of the marketization process of the firm's business place. The marketization process reflects a series of large-scale institutional changes, which significantly improve resource allocation efficiency and contribute 39% to total factor productivity. Our paper measures the marketization level through the Fangang index. The Fangang index was developed by Fangang, Wang Xiaolu, and Zhu Hengpeng and reflects the progress of each region in market-oriented reforms as much as possible. Because the calculation method is different before and after 2008, our paper uses the city rankings of the Fangang index as the marketization process. The higher a city's ranking, the better the marketization process.
  List style. Generally, firms choose how to go public based on their asset quality, which means that good firms prefer to go public through an IPO and poor firms prefer to go public through a shell listing [28]. Anderson et al. [29] divided family firms into two categories: “competition style” and “private benefits of control style.” The former kind of family firms focuses more on the firms' long-term strategy, and these firms initially wish to operate well in the long term, which could promote their investment efficiency. The latter kind of family firms cares more about self-interest, and the stakeholders and managers of such firms prefer immediate interests, which could decrease firms' investment efficiency. Thus, we consider “competition style” family firms to be good firms, for which the listing style is direct. “Private benefits of control style” family firms are poor firms that choose an indirect listing style. In this paper, the firms that choose the direct listing style take the value of 1, and those that choose the indirect listing style take the value of 0.
  Transparency level. This variable reflects the information asymmetry level of the family firm. Based on the literature, scholars believe that tracked analysts can disclose more detailed information about target firms. Thus, we use the natural logarithm of the number of analysts tracked to measure firms' transparency level.

#### 3.3.4. Control Variables

In this model, control is a vector for the control variables, which follow the literature on the determinants of investment efficiency [30–32]. These are the logarithm of total assets (Siz), the ratio of total debt to total assets (Lev), the cash flow from operating activities (Cas), the stock yearly return (Ret), firms' book value-to-market value ratio, return on assets (Roa), and firms' net profit growth rate (Dev).

We winsorize all data by 1%. The symbols and definitions of all variables are shown in Table 1.

## 4. Empirical Results

### 4.1. Statistical Description of the Data

The descriptive statistics of the variables used in this study are shown in Table 2. During the period under analysis, approximately 37.9% of family firms hired nonfamily managers, and 41% of family firms changed their controlling power.

### 4.2. The Main Regression (Family Exit and Investment Efficiency)

Table 3 shows the basic relationship between family exit and investment efficiency. The results in column 1 suggest that when family firms hire nonfamily managers, doing so decreases firms' investment efficiency. The interaction variable is 0.023, which is significant at the 1% level. The results in column 2 show that when family firms transfer the controlling power to nonfamily members, doing so also decreases investment efficiency; the interaction variable is 0.011 and significant at the 1% level.

### 4.3. The Market Reaction to Family Members' Punishment

The previous analysis shows that when family members hire nonfamily members or give up controlling power, doing so decreases firms' investment efficiency. This result implies that family members are very important to family firms. To test these findings, we determine the market reaction to family members' punishment.

Based on the previous literature, we use the CAR (cumulative abnormal return) to measure the market reaction. The calculation of the CAR is based on the market model, which is as follows:

(3) $$\begin{array}{c} R_{i,t}=\alpha_{i}+\beta_{i}R_{i,m}+\varepsilon_{i,t}, \end{array}$$

where *R*_*i*,*t*_ is the real rate of return, *R*_*i*,*m*_ is the market return in period *t*, and *ε*_*i*,*t* _ is a random error term. The regression of the equation above and parameter estimation are used to estimate *α*_*i*_ and *β*_*i*_. Then, assuming that *α*_*i*_ and *β*_*i*_ remain the same, we can obtain the abnormal return and cumulative abnormal return. The model is as follows:

(4) $$\begin{array}{c} {\text{AR}}_{i,t}=R_{i,t}-\alpha_{i}-\beta_{i}R_{i,m}, \end{array}$$

where AR_*i*,*t*_ is the abnormal return of stock *i* in period *t*, *R*_*i*,*t*_ is the real return of stock *i* in the period *t*, *R*_*i*,*m*_ is the market return in period *t*, and *α*_*i*_ and *β*_*i*_ is the estimation based on the market model. The CAR is the cumulative of AR_*i*,*t*_. The event window is three days before the punishment declaration date and three days after the punishment declaration date.

The results in Table 4 indicate that the market reaction changes (0.016) and is significant at the 5% level if family members are punished by the SEC. We conclude that family members are very important for family firms.

### 4.4. Investment Efficiency in Different Investment Levels

The literature divides investment into two categories: overinvestment and underinvestment. From the previous regression test, we know that family exit could decrease firms' investment efficiency. Furthermore, to obtain more detailed information about family exit and firms' investment efficiency, we want to know whether the effect could be the same under different investment levels. The different investment levels are defined by the residuals of Model (2); firms' investment level is high if the residual is positive, and vice versa.

Table 5 shows that family exit influences investment efficiency under a low investment level. Column (1) reveals that when family members hire nonfamily managers, doing so decreases investment efficiency, and this result is significant at the 1% level. Moreover, in column (2), the interaction variable is positive and significant at the 1% level. The results indicate that under a low investment level, the family exit will further reduce investment, thereby decreasing investment efficiency.

Table 6 presents the results of how family exit affects investment efficiency under a high investment level. In both columns (1) and (2), the interaction variable is negative and significant at the 5% and 1% levels, respectively. The results imply that family exit can increase firms' investment efficiency under high investment levels. The reason is that family members prefer long-term investment due to their family nature. Thus, a high investment level can offset the negative effect of family exit.

## 5. Moderating Effects

In this subsection, we examine the impact of moderators on the relationship between family exit and firms' efficiency at the meso level and micro level. We first investigate the moderating effect of the marketization level, which is considered the meso level. Then, we examine how firms' categories and information asymmetry affect the relationship between family exit and firms' efficiency, which is considered the micro level.

### 5.1. Investment Efficiency in Different Marketization Levels

The market environment is the general background of business operations, and there are region-level impact factors among firms' operating environments. Within the area of our sample, the marketization level is the main influencing factor in firms' operating ability. The marketization level could improve an area's competition level. Competition threatens the profit and even the survival of firms, which in turn requires firms to devote more attention and resources to deal with interfirm competition [33].

In this paper, if the area where a firm operates is developing fast or shows a growing development trend, we consider the area to have a better marketization level. We use the Fangang index to measure the marketization level. We test the relationship between family exit and firm investment efficiency under different marketization levels through the DID model as follows:

(5) $$\begin{array}{c} \text{Investment }{\text{Efficiency}}_{i}=\beta_{0}+\beta_{1}\text{Transfer}\times \text{Post}\times \text{Fangang}+\beta_{2}{\text{Controls}}_{i}+\theta_{i}, \end{array}$$

where the interaction variable Transfer × Post × Fangang is the key variable. If the key variable is significantly positive, the results indicate that the higher the Fangang index, the higher the firm's investment efficiency, and vice versa.

Table 7 presents the regression results. Line (1) is the situation of family members hiring nonfamily managers, and line (2) is family members giving up control power. From the table, we find that the interaction variable is negative and significant, and the results indicate that a higher marketization level could mitigate the relationship between family exit and firms' investment efficiency.

### 5.2. Investment Efficiency in Different List Styles

From previous studies, we know that family firms can be divided into two categories: “competition style” and “private benefits of control style” [29]. Generally, firms choose how to go public based on their asset quality, which means that good firms prefer to go public through an IPO and poor firms prefer to go public through a shell listing [28]. Thus, we consider the directing list method the “competition style” and consider the indirect listing method the “private benefits of control style.”

To test the relationship between family exit and investment efficiency under different firm categories, the DID model is as follows:

(6) $$\begin{array}{c} \text{Investment }{\text{Efficiency}}_{i}=\beta_{0}+\beta_{1}\text{Transfer}\times \text{Post}\times \text{List}+\beta_{2}{\text{Controls}}_{i}+\theta_{i}, \end{array}$$

where the interaction Transfer × Post × List is the key variable. We use firms' listing styles to measure the category of family firms. If a firm goes public directly, it is considered to have a “competition” style. If a firm goes public indirectly, it is considered to have a “private benefits of control” style.

Table 8 presents the regression results of family exit and firms' investment efficiency under different styles of firms. We find that the interaction variable in line (1) is positive but not significant. The interaction variable in line (2) is significantly positive, which means that “competition” style family firms have decreased investment efficiency. The results show that family firm categories have no significant influence on the relationship between families hiring outsider managers and firms' investment efficiency.

### 5.3. Investment Efficiency in Different Transparency Levels

Prior studies have suggested that information asymmetry is the main influencing factor in the efficiency of corporate investment [34]. Between corporate insiders and the capital market, investors must compete to obtain valuable information about firms' performance and future potential [18]. At the firm level, the transparency level could influence firms' information asymmetry; thus, we would like to test how family exit influences firms' investment efficiency.

Similar to previous studies, we also use a DID model to test the relationship between family exit and investment efficiency under different transparency levels.

(7) $$\begin{array}{c} \text{Investment }{\text{Efficiency}}_{i}=\beta_{0}+\beta_{1}\text{ Transfer}\times \text{Post}\times \text{Ana}+\beta_{2}{\text{Controls}}_{i}+\theta_{i}, \end{array}$$

where the key variable is the interaction variable. The regression results are presented in Table 9. We can see that the interaction variable in line (1) is positive but not significant, which means that the number of tracked analysts has no influence on the relationship between families hiring outsider managers and investment efficiency. However, the interaction variable in line (2) is significantly positive, which means that the number of tracked analysts decreases investment efficiency when family members give up their controlling power in the firm.

## 6. Conclusions

Researchers have argued about whether family or nonfamily firms are better from several perspectives. This study is based on the problem of family exit and discovers the economic consequence of family exit from the perspective of dynamic changes in family firms. Based on a panel data set of Chinese family firms from 2003 to 2019, we find that firms' investment efficiency decreases after family exit; in particular, we provide evidence that family members play important roles in family firm management. Then, we analyze several situations that can offset the negative effect. The results show that under a lower investment level, family exit decreases firms' investment efficiency, and vice versa. In an additional analysis, the marketization level increases firms' investment efficiency; other factors, such as firms' categories and transparency level, have no influence on the relationship between families hiring outsider managers and investment efficiency. However, when families give up controlling power, investment efficiency is decreased. In summary, our findings show that when a family exits from a family firm, doing so can influence the firm's investment efficiency.

## Figures and Tables

**Table 1:** Variable definitions.

Investment efficiency	Based on the research of Richardson [6], our paper establishes a model using the model residual to measure investment efficiency. The larger the absolute value of the residual, the lower the investment efficiency.
Tra1/2	Hiring nonfamily members, transfer1 takes the value of 1, and vice versa. Selling firms, transfer2 takes the value of 1, and vice versa.
Siz	The natural log of firms' total assets
Lev	The firms' leverage
Cas	The firms' operating net cash flow
Ret	The firms' stock yearly return
Tob	The firms' value
Rbm	The ratio of assets to market value
Roa	The firms' return on assets
Dev	The firms' net profit growth rate
Ana	The natural log of firms' analyst numbers

**Table 2:** Variable description.

Panel A: dummy variable description					
Variable	Obs	Mean		Std. dev.	
Tra1	6,842	0.379		0.485	
Tra2	6,842	0.410		0.796	

Panel B: continuous variables description					
Variable	Obs	Mean	Std. dev.	Min	Max

Investment efficiency	6,842	0.100	0.088	0.002	0.442
Siz	6,842	21.755	1.183	18.475	24.788
Lev	6,842	3.250	3.081	0.424	21.925
Cas	6,838	0.154	0.127	0.002	0.764
Ret	6,842	0.252	0.758	−0.714	3.172
Tob	6,835	0.030	0.086	−0.556	0.226
Roa	6,607	0.572	0.239	0.114	1.096
Dev	6,842	0.379	0.485	0.002	0.442

**Table 3:** Regression of investment efficiency and family exit.

	(1)	(2)
	Investment efficiency	Investment efficiency
Tra1 ^∗^ post	0.023^*∗∗∗*^	
	(10.37)	
Tra2 ^∗^ post		0.011^*∗∗∗*^
		(8.32)
Size	−0.009^*∗∗∗*^	−0.009^*∗∗∗*^
	(−6.81)	(−6.86)
Lev	−0.002^*∗∗∗*^	−0.002^*∗∗∗*^
	(−5.21)	(−5.39)
Cas	−0.005	−0.006
	(−0.61)	(−0.63)
Ret	0.004^*∗*^	0.003
	(1.79)	(1.38)
Dev	−0.073^*∗∗∗*^	−0.077^*∗∗∗*^
	(−11.02)	(−11.63)
Roa	−0.075^*∗∗∗*^	−0.080^*∗∗∗*^
	(−5.87)	(−6.22)
Yea	Control	Control
Ind	Control	Control
Are	Control	Control
Con	0.344^*∗∗∗*^	0.360^*∗∗∗*^
	(11.93)	(12.48)
*N*	6,596	6,596

*t* statistics are in parentheses. ^*∗*^*p* < 0.10, ^*∗∗*^*p* < 0.05, and ^*∗∗∗*^*p* < 0.01.

**Table 4:** Market reaction on family punishment.

	(1)
	CAR
Punish	0.016^*∗∗*^
	(2.29)
Lev	−0.001
	(−0.99)
Size	0.001
	(0.17)
Roa	0.005^*∗∗∗*^
	(3.79)
Tob	0.001
	(1.01)
Ind	Control
Are	Control
Yea	Control
Con	0.0964
	(1.37)
*N*	1305

*t* statistics are in parentheses. ^*∗*^*p* < 0.10, ^*∗∗*^*p* < 0.05, and ^*∗∗∗*^*p* < 0.01.

**Table 5:** Low investment level.

	(1)	(2)
	Investment efficiency	Investment efficiency
Tra1 ^∗^ post	0.034^*∗∗∗*^	
	(18.68)	
Tra2 ^∗^ post		0.017^*∗∗∗*^
		(15.74)
Size	−0.070^*∗∗∗*^	−0.070^*∗∗∗*^
	(−51.14)	(−50.49)
Lev	−0.004^*∗∗∗*^	−0.004^*∗∗∗*^
	(−12.66)	(−12.93)
Cas	−0.011	−0.011
	(−1.62)	(−1.54)
Ret	0.007^*∗∗∗*^	0.005^*∗∗∗*^
	(3.76)	(2.90)
Dev	−0.005	−0.012^*∗∗*^
	(−0.88)	(−1.99)
Roa	0.009	0.004
	(0.97)	(0.41)
Yea	Control	Control
Ind	Control	Control
Are	Control	Control
Con	1.580^*∗∗∗*^	1.601^*∗∗∗*^
	(56.35)	(56.43)
*N*	3,903	3,903

*t* statistics are in parentheses. ^*∗*^*p* < 0.10, ^*∗∗*^*p* < 0.05, and ^*∗∗∗*^*p* < 0.01.

**Table 6:** High investment level.

	(1)	(2)
	Investment efficiency	Investment efficiency
Tra1 ^∗^ post	−0.009^*∗∗*^	
	(−2.27)	
Tra2 ^∗^ post		−0.007^*∗∗∗*^
		(−2.58)
Size	0.038^*∗∗∗*^	0.038^*∗∗∗*^
	(16.31)	(16.33)
Lev	0.003^*∗∗∗*^	0.003^*∗∗∗*^
	(4.24)	(4.23)
Cas	−0.047^*∗∗∗*^	−0.047^*∗∗∗*^
	(−2.68)	(−2.68)
Ret	0.015^*∗∗∗*^	0.015^*∗∗∗*^
	(3.69)	(3.78)
Dev	−0.013	−0.011
	(−1.18)	(−1.01)
Roa	0.046	0.050
	(1.40)	(1.51)
Yea	Control	Control
Ind	Control	Control
Are	Control	Control
Con	−0.759^*∗∗∗*^	−0.761^*∗∗∗*^
	(−12.63)	(−12.66)
*N*	2693	2693

*t* statistics are in parentheses. ^*∗*^*p* < 0.10, ^*∗∗*^*p* < 0.05, and ^*∗∗∗*^*p* < 0.01.

**Table 7:** OLS regression in different marketization levels.

	(1)	(2)
	Investment efficiency	Investment efficiency
Tra1 ^∗^ post ^∗^ Fangang	−0.017^*∗∗∗*^	
	(−6.46)	
Tra2 ^∗^ post ^∗^ Fangang		−0.030^*∗∗∗*^
		(−8.91)
Size	0.011^*∗∗∗*^	0.011^*∗∗∗*^
	(3.02)	(3.01)
Lev	0.004^*∗∗∗*^	0.004^*∗∗∗*^
	(3.38)	(3.43)
Cas	0.014	0.011
	(0.58)	(0.46)
Ret	−0.058^*∗∗∗*^	−0.058^*∗∗∗*^
	(−10.12)	(−10.18)
Rbm	−0.398^*∗∗∗*^	−0.399^*∗∗∗*^
	(−21.74)	(−22.02)
Roa	−0.096^*∗*^	−0.084
	(−1.77)	(−1.57)
Dev	0.001^*∗∗∗*^	0.001^*∗∗∗*^
	(6.35)	(6.40)
Yea	Control	Control
Ind	Control	Control
_con	0.198^*∗∗∗*^	0.202^*∗∗∗*^
	(2.76)	(2.85)
*N*	3,146	3,146

*t* statistics are in parentheses. ^*∗*^*p* < 0.10, ^*∗∗*^*p* < 0.05, and ^*∗∗∗*^*p* < 0.01.

**Table 8:** OLS regression in different list levels.

	(1)	(2)
	Investment efficiency	Investment efficiency
Tra1 ∗ post ∗ list	0.011	
	(1.34)	
Tra2 ∗ post ∗ list		0.041^*∗∗∗*^
		(3.48)
Size	0.003	0.003
	(0.74)	(0.79)
Lev	0.003^*∗∗*^	0.003^*∗∗*^
	(2.52)	(2.55)
Cas	−0.035	−0.037
	(−1.26)	(−1.34)
Ret	−0.076^*∗∗∗*^	−0.076^*∗∗∗*^
	(−9.99)	(−9.94)
Rbm	−0.445^*∗∗∗*^	−0.445^*∗∗∗*^
	(−20.92)	(−21.01)
Roa	−0.068	−0.064
	(−1.04)	(−0.98)
Dev	0.001^*∗∗∗*^	0.001^*∗∗∗*^
	(6.68)	(6.56)
Yea	Control	Control
Ind	Control	Control
Are	Control	Control
Con	0.346^*∗∗∗*^	0.337^*∗∗∗*^
	(3.92)	(3.83)
*N*	2,297	2,297

*t* statistics are in parentheses. ^*∗*^*p* < 0.10, ^*∗∗*^*p* < 0.05, and ^*∗∗∗*^*p* < 0.01.

**Table 9:** OLS regression in different transparency levels.

	(1)	(2)
	Investment efficiency	Investment efficiency
Tra1 ∗ post ∗ Ana	0.012	
	(1.36)	
Tra2 ∗ post ∗ Ana		0.038^*∗∗∗*^
		(3.19)
Size	0.010^*∗∗∗*^	0.009^*∗∗*^
	(2.59)	(2.45)
Lev	0.003^*∗∗∗*^	0.003^*∗∗∗*^
	(3.10)	(3.07)
Cas	0.009	0.008
	(0.37)	(0.32)
Ret	−0.059^*∗∗∗*^	−0.059^*∗∗∗*^
	(−10.32)	(−10.31)
Rbm	−0.407^*∗∗∗*^	−0.408^*∗∗∗*^
	(−22.14)	(−22.26)
Roa	−0.111^*∗∗*^	−0.109^*∗∗*^
	(−2.05)	(−2.02)
Dev	0.001^*∗∗∗*^	0.001^*∗∗∗*^
	(6.58)	(6.47)
Yea	Control	Control
Ind	Control	Control
Are	Control	Control
Con	0.246^*∗∗∗*^	0.259^*∗∗∗*^
	(3.33)	(3.54)
*N*	3,148	3,148

*t* statistics are in parentheses. ^*∗*^*p* < 0.10, ^*∗∗*^*p* < 0.05, and ^*∗∗∗*^*p* < 0.01.

## Data Availability

The data used are available within the article.
